The article "Effect of Intensive Psychological Care on Patients with Benign Breast Lumps after Mammotome-Assisted Tumor Resection" was retracted in 2023. Reasons: signs of a paper mill; compromised peer review; unreliable results or conclusions.

# Effect of Intensive Psychological Care on Patients with Benign Breast Lumps after Mammotome-Assisted Tumor Resection

**DOI:** 10.1155/2022/9054266

**Published:** 2022-06-24

**Authors:** Ping Xu, Ronghua Xu, Qingfeng Yang, Hongfeng Zhu

**Affiliations:** ^1^Department of Comprehensive Surgery, Anhui Province Maternal &Child Health Hospital West Hospital, Hefei, China; ^2^Department of Nursing, Anhui Province Maternal &Child Health Hospital, Hefei, China; ^3^Department of Obstetrics, Anhui Province Maternal &Child Health Hospital, Hefei, China

## Abstract

**Objective:**

The aim of the study was to evaluate the effect of intensive psychological care on patients with benign breast lumps after Mammotome-assisted tumor resection.

**Methods:**

A total of 160 patients with benign breast lumps diagnosed and treated in our hospital between May 2019 and January 2021 were recruited and divided into a study group (*n* = 80) and a control group (*n* = 80) via the random number table method. All patients received Mammotome-assisted tumor resection. Patients in the control group received conventional nursing, and those in the study group received intensive psychological care. The outcome measure included quality of life of patients, psychological states, treatment compliance, and nursing satisfaction.

**Results:**

The differences in the Functional Assessment of Cancer Therapy-General (FACT-G) scores, self-rating anxiety scale (SAS) scores, Hamilton Depression Rating Scale (HAMD) scores, and Morisky scores between the two groups were not significant before the intervention (*p* > 0.05). The FACT-G scores improved in both groups after the intervention, with higher results in the study group than those in the control group (*p* < 0.05). Patients in the study group showed a significantly greater reduction in the SAS and HAMD scores than those in the control group (*p* < 0.05). Intensive psychological care used in the study group resulted in significantly higher compliance scores in the body mass control, medication compliance, exercise compliance, and dietary compliance versus conventional care for the control group (*p* < 0.05).

**Conclusion:**

Intensive psychological care provides satisfactory outcomes in patients with benign breast lumps after Mammotome-assisted tumor resection. It effectively improves the quality of life of patients, relieves their negative emotions, and strengthens treatment compliance and patient satisfaction, which shows good potential for clinical promotion.

## 1. Introduction

Breast cancer [1, 2] is the result of the uncontrolled proliferation of breast epithelial cells under the influence of various carcinogenic factors. Its clinical manifestations are mostly breast nodules, bleeding nipples, and enlarged axillary lymph nodes. Advanced breast cancer may develop distant metastases, leading to multiorgan damage and risk of death [3]. Epidemiological statistics show that the prevalence of breast cancer ranks first among malignant tumors in women, accounting for 24.2%. Benign breast lumps [4] are commonly seen in young women, with fibroadenomas being the most frequent. Excessive oestrogen stimulation, an imbalance between oestrogen and progesterone secretion, or local breast tissue hypersensitivity to oestrogen promotes abnormal proliferation of epithelial and mesenchymal components of the breast and is associated with the formation of benign breast masses. Genetic factors for benign breast masses have also been reported as previous studies have found genetic abnormalities in 20–30% of patients with fibroadenoma of the breast [5, 6]. Moreover, it has been indicated that the risk of malignant transformation of benign breast lumps is 2–3 times higher compared with the normal population, which seriously affects the life and health of patients [7]. Surgery is the mainstay of treatment for breast tumors, and Mammotome-assisted tumor resection is an effective surgical approach. During Mammotome-assisted tumor resection, a small hole of about 3 mm was pierced in a hidden place such as the axilla or areola, and the lump was located and resected using the Mammotome vacuum-assisted breast biopsy system, with benefits such as small wound, less pain, shorter hospital stays, and faster postoperative recovery [8, 9]. Most patients suffer from varying degrees of psychological problems and negative emotions due to a lack of awareness of the disease, which hinders the smooth implementation of surgery and recovery, thus seriously affecting the quality of life and psychological well-being. Therefore, postoperative care to alleviate patients' negative emotions and encourage active treatment cooperation is essential. Intensive psychological care provides patients with different forms and degrees of psychological aid and supports to induce a sense of psychological satisfaction and security, thus relieving their psychological stress and negative emotions. However, there is a dearth of studies on the effect of intensive psychological care on patients with benign breast lumps after Mammotome-assisted tumor resection [10]. To this end, the aim of this study was to evaluate the impact of intensive psychological care on patients with benign breast masses after Mammotome-assisted tumor resection and to provide further data to support related studies.

The article "Effect of Intensive Psychological Care on Patients with Benign Breast Lumps after Mammotome-Assisted Tumor Resection" was retracted in 2023. Reasons: signs of a paper mill; compromised peer review; unreliable results or conclusions.

## 2. Materials and Methods

### 2.1. Participants

A total of 160 patients with benign breast lumps diagnosed and treated in our hospital between May 2019 and January 2021 were recruited, and all eligible patients were female, aged 30–68 (46.83 ± 6.17) years. They were assigned to a study group (*n* = 80) and a control group (*n* = 80) via a random number table method. All patients received Mammotome-assisted tumor resection. Patients in the control group received conventional nursing, and those in the study group received intensive psychological care.

### 2.2. Inclusion and Exclusion Criteria

The inclusion criteria were as follows: (1) diagnosis of a benign breast tumor in accordance with the clinical diagnostic criteria of the International Federation of Obstetrics and Gynaecology [11]; (2) undergoing Mammotome adjuvant tumor resection at our institution; and (3) patients who provided written informed consent were included in the study.

The exclusion criteria were as follows: (1) severe cardiac, hepatic, or renal dysfunction or organic pathology; (2) psychiatric illness or unconsciousness; (3) pregnancy and lactation; and (4) patients with contraindications to treatment.

### 2.3. Treatment Methods

All patients underwent Mammotome-assisted tumor resection. The location, size, and depth of the lesion were accurately located preoperatively. Patients were placed in a supine position with lateral shoulder elevation. After routine disinfection, 1–2 drops of epinephrine and 20 ml of 0.5% lidocaine were injected into the selected prepuncture site. An incision of approximately 3 mm was made at the injection site, and the rotary blade was inserted, moved underneath the lump, and pressed against the bottom of the lump under ultrasound guidance. The position of the blade slot was adjusted to align the lesion, followed by rotary resection and aspiration of the lesion. After the lesion was excised, the residual blood was removed by vacuum aspiration. The wound was covered with sterile gauze without sutures, and local compression was applied to the original lesion for more than 10 minutes to ensure good hemostasis, followed by compression bandaging with an elastic bandage.

Patients in the control group received routine care, including health education on tumor knowledge, preoperative examination, intraoperative adjuvant physician, vital signs monitoring, and postoperative basic care.

Patients in the study group received intensive psychological care:

1. Preoperative care: psychological status assessment of patients upon admission and active communication was performed to understand the causes of negative emotions and ensure effective preoperative preparation. The patients were also educated about the cause, treatment, and prognosis of the disease as well as the need and benefits of surgical treatment to reduce their anxiety and fear. Soothing and decompression methods such as playing soothing music may help patients relax.
2. Intraoperative care: the temperature and humidity in the operating room should be properly managed to ensure a comfortable external environment. Nursing staff talked slowly and gently with patients during the operation to guide them to maintain a positive and stable psychological state and avoid stress reactions.
3. Postoperative care: the patients were informed of the surgical results immediately after they recovered from anesthesia and visited frequently for close observation of their status to establish a good nurse-patient relationship. The family members of the patients were also instructed to provide the patients with encouragement and support to enhance their life attitudes. Cognitive therapy was used to help the patients understand the correlation of disease with negative emotions, and biofeedback therapy instruments were used to collect physiological signals of the patients, which contribute to enhancing the self-regulation and treatment compliance of patients.

The article "Effect of Intensive Psychological Care on Patients with Benign Breast Lumps after Mammotome-Assisted Tumor Resection" was retracted in 2023. Reasons: signs of a paper mill; compromised peer review; unreliable results or conclusions.

### 2.4. Outcome Measures

1. Quality of life [12]: the Functional Assessment of Cancer Therapy - General (FACT-G) was used to evaluate the quality of life in four aspects: emotional function, cognitive function, social function, and physical function, using a scale of 0–4 points, with a total of 27 items and a total score of 108 points.
2. Negative emotions [13]: the Self-Rating Anxiety Scale (SAS) and the Hamilton Depression Rating Scale (HAMD) were used to assess the negative emotions of patients. The SAS scale consisted of 20 items with a total score of 100 points, with 50–70 points being mild anxiety, 71–90 points being moderate anxiety, and >90 points being severe anxiety. The higher the score, the more severe the anxiety. The HAMD scale consists of 24 items and was scored on a scale of 0–4 points, and the higher the score, the more severe the depression.
3. Compliance [14]: the Morisky compliance scale was used to evaluate the patients' compliance with treatment before and after nursing intervention in four aspects: medication compliance, body mass control, dietary compliance, and exercise compliance, with a full score of 50 points, with higher scores indicating higher compliance.
4. Satisfaction: the “Nursing Satisfaction Questionnaire” (including the attitude of healthcare personnel, efficiency of care, and disease education) created by our hospital was divided into four levels (highly satisfied, satisfied, less satisfied, and dissatisfied) to understand the satisfaction of patients in both groups.

The article "Effect of Intensive Psychological Care on Patients with Benign Breast Lumps after Mammotome-Assisted Tumor Resection" was retracted in 2023. Reasons: signs of a paper mill; compromised peer review; unreliable results or conclusions.

### 2.5. Statistical Analysis

GraphPad Prism 8 software was used to plot the graphics, and SPSS22.0 software was used for data analyses. The count data are expressed as rates (*n* (%)) and analyzed using the chi-square test, and the measurement data are expressed as the mean ± standard deviation and analyzed using Student's *t*-test. Statistically significant results were defined as *p* < 0.05.

## 3. Results

### 3.1. Patient Characteristics

There were 80 patients in the control group, aged 30–65 (46.55 ± 6.23) years, with a disease duration of 0.8–4.0 (2.02 ± 0.27), a mean tumor diameter of 0.6–2.8 cm (1.28 ± 0.41) cm; there were 35 cases of breast hyperplasia, 38 cases of breast fibroids, and 7 cases of other in terms of pathological types. There were 80 patients in the control group, aged 32–68 (46.98 ± 5.89) years, with a disease duration of 1.0–3.9 (1.98 ± 0.35), a mean tumor diameter of 0.5–2.5 cm (1.17 ± 0.39) cm; there were 33 cases of breast hyperplasia, 36 cases of breast fibroids, and 11 cases of other in terms of pathological types. There were no significant differences in the baseline patient characteristics between the two groups (*p* > 0.05) (Table 1).

### 3.2. Quality of Life

No significant difference was found in the FACT-G scores between the two groups before the intervention (*p* > 0.05). The FACT-G scores improved in both groups after the intervention, with higher results in the study group (87.21 ± 5.57) than those in the control group (64.84 ± 6.28) (*p* < 0.05) (Table 2).

### 3.3. Negative Emotions

There was no statistically significant difference in the SAS and HAMD scores between the two groups of patients before the intervention (*p* > 0.05). After the intervention, patients in the study group showed a significantly greater reduction in the SAS and HAMD scores (32.15 ± 3.18, 33.08 ± 4.11) than those in the control group (51.51 ± 4.54, 40.36 ± 5.65) (*p* < 0.05) (Table 3).

### 3.4. Treatment Compliance

The differences in the Morisky scores between the two groups did not come up to the statistical standard before intervention (*p* > 0.05). After the intervention, intensive psychological care used in the study group resulted in significantly higher compliance scores in the body mass control, medication compliance, exercise compliance, and dietary compliance (39.67 ± 2.24, 41.92 ± 2.41, 42.01 ± 2.08, and 43.88 ± 3.12) versus conventional care for the control group (28.17 ± 3.21, 29.87 ± 2.65, 30.79 ± 3.18, and 33.25 ± 4.11) (*p* < 0.05) (Figure 1).

### 3.5. Nursing Satisfaction

In the control group, there were 26 (32.50%) cases of highly satisfied, 35 (43.75%) cases of satisfied, 11 (13.75%) cases of less satisfied, and 8 (10.00%) cases of dissatisfied. In the study group, there were 33 (41.25%) cases of highly satisfied, 45 (56.25%) cases of satisfied, 1 (1.25%) case of less satisfied, and 1 (1.25%) case of dissatisfied (Table 4).

The article "Effect of Intensive Psychological Care on Patients with Benign Breast Lumps after Mammotome-Assisted Tumor Resection" was retracted in 2023. Reasons: signs of a paper mill; compromised peer review; unreliable results or conclusions.

## 4. Discussion

The incidence of breast cancer is increasing year by year and has leapt to the top of the list of malignant tumors in women, estimated to be close to 0.03%, i.e., close to 3 per 10,000 people worldwide [15]. Breast cancer is more common in women between the ages of 40 and 60 and is relatively uncommon in women younger than 35 years [16]. Breast cancer is now considered to be multifactorial. Family history is a high-risk factor for breast cancer; early menarche, late menopause, and benign breast disease are also risk factors; chronic use of exogenous oestrogens or alcohol and depression are also risk factors, and genetic mutations may also play an important role [17, 18]. Biopsied open surgery of clinical breast lesions has been the conventional method in the past, which can completely remove the mass and provide sufficient tissue volume for pathological diagnosis [19]. However, it may leave obvious scars, affect the beauty of the breasts, and cause great mental stress and psychological burden to female friends [20].

The Mammotome system, developed by Johnson & Johnson, is the most advanced minimally invasive biopsy system available. It consists of two main devices: a rotary cutter and a vacuum suction pump, which allow repeated cutting of suspicious breast lesions to obtain histological specimens of the breast, providing more and better methods for the detection and diagnosis of breast cancer, as well as a technical basis for minimally invasive excision of benign tumors [21, 22]. Ultrasound-guided breast puncture biopsy and the complete excision system can diagnose most breast lesions. Mammotome allows for minimally invasive biopsy of diseased breast tissue under ultrasound guidance, while complete excision of some benign tumors can be performed under ultrasound guidance [23]. Mammotome is the gold standard for biopsy of calcified lesions and is uniquely designed to make biopsies easier and more definitive [22, 23]. Mammotome is designed to be used in conjunction with a molybdenum-targeting system to its fullest advantage. The needle can be rotated 360 degrees to ensure large, continuous specimens are obtained, and there are two types of localised biopsies, both firing and nonfiring, making it possible to biopsy deep lesions and smaller breasts with greater diagnostic accuracy than previous fine and coarse needle punctures [24].

Psychological care refers to the application of psychological methods and practices to achieve a positive psychological impact on patients [25], and intensive psychological care provides patients with different forms and degrees of psychological help and support [26, 27]. Traditional mastectomy can leave scars and lead to negative emotions, and studies have shown that 98% of breast cancer patients experience anxiety and depression [3, 28]. Mammotome-assisted tumor resection is characterised by precise positioning, ease of operation, and small incisions and being combined with intensive psychological care can alleviate patients' postoperative moods [29, 30]. The results of the present study showed that intensive psychological care resulted in significantly higher FACT-G scores, higher treatment compliance, and lower SAS and HAMD scores versus conventional care (*p* < 0.05), indicating that intensive psychological care benefits the quality of life and treatment compliance of patients by mitigating their negative emotions. Presumably, the reason can be that intensive psychological care enhances patients' understanding of the disease and the surgery to reduce their fear and foster a positive treatment attitude, which contributes to a successful surgery. In addition, intraoperative reassurance helps patients maintain a stable physical state and increase surgical tolerance, while postoperative psychological support alleviates negative postoperative emotions and encourages patients to communicate with others to achieve emotional release [31]. Moreover, patients in the study group showed a significantly higher nursing satisfaction (97.50%) than those in the control group (76.25%) (*p* < 0.05), suggesting that intensive psychological care is effective in enhancing the quality of life of patients and alleviating their negative emotion [32, 33]. This result is in concordance with the research results by Jimmy Kim et al., which reported that psychological care was associated with higher nursing satisfaction in breast cancer patients after surgical resection.

The article "Effect of Intensive Psychological Care on Patients with Benign Breast Lumps after Mammotome-Assisted Tumor Resection" was retracted in 2023. Reasons: signs of a paper mill; compromised peer review; unreliable results or conclusions.

However, our experiments also have certain flaws. The first is the chance caused by the small sample size. Second, we need a large number of return visits to determine long-term efficacy. In addition, Mammotome's use in other diseases (such as breast hyperplasia and malignancy) is less studied, and further clinical trials are needed. Finally, minimal residual disease caused by incomplete resection may not always be detected by ultrasound, and further studies are needed to determine the prognostic effect.

## 5. Conclusion

Intensive psychological care provides satisfactory outcomes in patients with benign breast lumps after Mammotome-assisted tumor resection. It effectively improves the quality of life of patients, relieves their negative emotions, and strengthens treatment compliance and patient satisfaction, which shows good potential for clinical promotion.

## Figures and Tables

**Figure 1:** Morisky scores. The symbol ^*∗*^indicates that there is a statistically significant difference (*p* < 0.05) between the two groups. (a) Body mass control; (b) medication compliance; (c) exercise compliance; (d) dietary compliance.

**Table 1:** Patient characteristics ($\bar{x}\pm s$$\bar{\text{x}}$).

Group	*n*	Age (year)		Course of disease (year)		Tumor diameter (cm)		Pathological types		
		Mean	Range	Mean	Range	Mean	Range	Breast hyperplasia	Breast fibroids	Other
Control	80	46.55 ± 6.23	30–65	2.02 ± 0.27	0.8–4.0	1.28 ± 0.41	0.6–2.8	35	38	7
Study	80	46.98 ± 5.89	32–68	1.98 ± 0.35	1.0–3.9	1.17 ± 0.39	0.5–2.5	33	36	11
*T*	—	0.287	—	0.361	—	0518	—	—	—	—
*p* value	—	0.787	—	0.728	—	0.596	—	—	—	—

**Table 2:** FACT-G scores ($\bar{x}\pm s$).

Group	*n*	Before intervention	After intervention
Control	80	43.28 ± 5.28	64.84 ± 6.28^*∗*^
Study	80	43.17 ± 5.65	87.21 ± 5.57^*∗*^
*T*	—	0.053	12.987
*p* value	—	0.958	<0.001

*Note.* The symbol *∗* indicates a statistically significant difference (*p* < 0.05) in the comparison between before and after treatment within the same group.

**Table 3:** SAS and HAMD scores ($\bar{x}\pm s$$\bar{\text{x}}$).

Group	*n*	SAS		HAMD	
		Before intervention	After intervention	Before intervention	After intervention
Control	80	66.83 ± 4.96	51.51 ± 4.54*∗*	53.53 ± 6.21	40.36 ± 5.65*∗*
Study	80	66.74 ± 5.17	32.15 ± 3.18*∗*	53.45 ± 6.08	33.08 ± 4.11*∗*
*t*	—	0.327	13.695	0.355	11.081
*p* value	—	0.798	<0.001	0.732	<0.001

*Note.* The symbol *∗* indicates a statistically significant difference (*p* < 0.05) in the comparison between before and after treatment within the same group.

**Table 4:** Nursing satisfaction (%).

Group	*n*	Highly satisfied	Satisfied	Less satisfied	Dissatisfied	Total satisfaction
Control	80	26 (32.50)	35 (43.75)	11 (13.75)	8 (10.00)	61 (76.25)
Study	80	33 (41.25)	45 (56.25)	1 (1.25)	1 (1.25)	78 (97.50)
*x* ^2^	—			8.624		
*p* value	—			0.001		

## Data Availability

No data were used to support this study.
